The article "Efficacy of Different Preemptive Analgesia on Postoperative Analgesia, Oxidative Stress, and Inflammatory Response after Gynecological Laparoscopic Surgery" was retracted in 2023. Reasons: unreliable results or conclusions; concerns about the data; concerns about the peer review; concerns about the citations.

# Efficacy of Different Preemptive Analgesia on Postoperative Analgesia, Oxidative Stress, and Inflammatory Response after Gynecological Laparoscopic Surgery

**DOI:** 10.1155/2021/4233716

**Published:** 2021-10-29

**Authors:** Chengcheng Sun, Qinghua Yang, Chenyu Wang, Jianyi Zhao, Ming Dai

**Affiliations:** ^1^Department of Anesthesiology, Yiwu Central Hospital, Yiwu, Zhejiang 322000, China; ^2^Department of Anorectal Surgery, Yiwu Central Hospital, Yiwu, Zhejiang 322000, China; ^3^Department of Anesthesiology, Changshan County People's Hospital, Quzhou, Zhejiang 324200, China

## Abstract

**Objective:**

To observe and compare the analgesic effects of oxycodone, pentazocine, and ketorolac tromethamine pre-emptive analgesia on gynecological laparoscopic patients after operation and the effects on oxidative stress and inflammatory reaction.

**Methods:**

A total of 64 patients who underwent elective gynecological laparoscopic surgery in Yiwu Central Hospital from June 2019 to December 2020 were randomly divided into four groups (*n* = 16). Before anesthesia induction, oxycodone (group A), pentazocine (group B), ketorolac tromethamine (group C), and normal saline (group D) were, respectively, administered. Patients' mean arterial pressure (MAP) and heart rate (HR) changes, visual analogue scale (VAS), Bruggemann comfort scale (BCS), serum tumor necrosis factor-*α* (TNF-*α*), interleukin-6 (IL-6), C-reactive protein (CRP), blood glucose (CLU), serum cortisol level, postoperative adverse reactions, and additional analgesia were recorded at each time point.

**Results:**

The MAP levels of T2 (immediate intubation), T3 (immediate catheter removal), and T4 (5 min after catheter removal) in the four groups were higher than those of T1 (quiescent state), and the HR levels T2, T3, and T4 were lower than those of T1 (*P* < 0.05). The MAP and HR levels of T2, T3, and T4 in patients of groups A, B, and C were lower than those of group D in the same period (*P* < 0.05). The VAS and BCS scores of groups A, B, and C at 1, 6, 12, and 24 h after operation were better than those of group D at the same time, and the scores of group A at 1 h and 6 h after operation were better than those of groups B and C at the same time (*P* < 0.05). The levels of serum TNF-*α*, IL-6, and CRP in the four groups of patients at 6, 12, and 24 h after operation were higher than those before operation, but those in groups A, B, and C were lower than those in group D, and those in group A were higher than those in groups B and C at 12 h and 24 h after operation (*P* < 0.05). The CLU and serum cortisol levels in the four groups were significantly higher at 6, 12, and 24 h after operation, but those in groups A, B, and C were lower than those in group D, and those in group A were lower than those in groups B and C at 6 and 12 h after operation (*P* < 0.05). There was no significant difference in the incidence of adverse reactions within 24 h between the four groups (*P* > 0.05). The incidence of additional analgesia in groups A, B, and C was lower than that in group D (*P* < 0.05).

**Conclusion:**

Oxycodone, pentazocine, and ketorolac tromethamine are effective and safe in inhibiting postoperative pain and the generation of inflammatory factors and relieving inflammatory state in gynecological laparoscopic pre-emptive analgesia. Oxycodone has better postoperative analgesic effect because it can effectively alleviate stress reaction.

## 1. Introduction

Laparoscopic surgery is a minimally invasive surgery commonly used in gynecology in recent years. It can be used to remove space-occupying lesions of the uterus and ovary and even clean the lymph nodes of malignant tumor. Compared with laparotomy, it has the advantages of less damage and rapid recovery. It has gradually replaced laparotomy, and its proportion in the field of gynecology has increased significantly [1]. However, postoperative patients still have to endure the pain caused by pneumoperitoneum, surgical incision, and uterine and accessory trauma. Even the main complications of injury are postoperative incision pain and visceral pain. If there is no effective treatment for pain, acute pain may develop into chronic pain [2]. Injuries such as surgical trauma can stimulate the neuroendocrine system, increase the secretion level of catecholamine in the body, stimulate the systemic stress response, and increase the level of proinflammatory cytokines, resulting in hyperalgesia in the nervous system of the body [3]. Therefore, in order to reduce or eliminate pain caused by injury during clinical anesthesia, analgesic measures should be taken before the injury acts on the body. In recent years, pre-emptive analgesia has been widely used in clinical anesthesia to prevent central and peripheral nerve hyperalgesia and reduce the level of synthesis and release of proinflammatory factors in the body, so as to better improve the postoperative inflammatory response and effectively reduce the postoperative pain [4]. Effective preemptive analgesia is very important for prognosis and rehabilitation of patients after gynecological laparoscopy.

Opioids and nonsteroidal drugs are commonly used as preemptive analgesics in gynecological surgery. Oxycodone is a semisynthetic derivative of opioid alkaloids. It is a pure opioid double-receptor agonist. It can reduce the synthesis of inflammatory cytokines by decreasing the content of cyclic adenosine monophosphate in cells. It has the advantages of rapid effect, strong and durable analgesic effect, stable hemodynamics, and low incidence of postoperative nausea and vomiting. It is mainly used for cancer pain treatment and postoperative analgesia [5, 6]. Pentazocine, also known as Zhentongxin, is an opioid analgesic like oxycodone and morphine. Its mechanism is different from that of morphine. Its respiratory depression, nausea and vomiting, and other side effects are less than morphine. In recent years, pentazocine has been widely used for postoperative analgesia and cancer analgesia [7]. Ketorolac tromethamine belongs to nonsteroidal anti-inflammatory drugs. Unlike fenic acids, it has no dependence on opioids. It has antipyretic, anti-inflammatory, and highly analgesic effects. It is metabolized into ketorolac in the human body to exert biological effects, which is often used for the treatment of acute pain after surgery [8]. The purpose of this study was to observe and compare the analgesic effects of oxycodone, pentazocine, and tromethamine on gynecological laparoscopic surgery and their effects on oxidative stress level and inflammatory factors after surgery. The report reads as follows.

## 2. Information and Methods

### 2.1. General Information

From June 2019 to December 2020, 64 patients who underwent elective gynecological laparoscopic surgery in Yiwu Central Hospital were randomly divided into four groups, with 16 patients in each group. The surgical methods included laparoscopic myomectomy in 21 patients, laparoscopic ovarian cyst stripping in 6 patients, laparoscopic salpingo-mesenteric cyst resection in 4 patients, laparoscopic bilateral tubal ligation in 8 patients, laparoscopic endometriosis lesion resection in 6 patients, and laparoscopic salpingectomy in 19 patients. Before anesthesia induction, oxycodone (group A), pentazocine (group B), ketorolac tromethamine (group C), and normal saline (group D) were, respectively, administered. The inclusion criteria were as follows: American Association of Anesthesiologists (ASA) grades I-II, no nonsteroidal anti-inflammatory drugs were taken within 3 days before operation, no use of analgesics within 1 week prior to surgery, no monoamine oxidase inhibitor was taken 15 days before surgery, and no history of anesthetic allergy. The exclusion criteria were as follows: patients with combined asthma history, patients with a history of severe ulcers, patients with combined medical history of hypertension, nervous system diseases, and mental diseases, and people who are allergic to the drugs used in the study. The study was approved by the Ethics Committee of our hospital, and the informed consent form was signed by the patients and their families.

### 2.2. Anesthesia Methods

Patients were deprived of food and water 8 h before operation. No medications were used before the operation. After entering the operating room, the peripheral venous channel was opened, and the fluid replacement rate was controlled at 10 mL/(kg h). Vital signs were continuously monitored: heart rate (HR), blood pressure (BP), and oxygen saturation (SpO_2_). All the patients were given general intravenous anesthesia after intravenous induction and intubation. Before anesthesia induction, oxycodone hydrochloride injection (0.1 mg/kg) was intravenously injected in group A, pentazocine injection (0.2 mg/kg) was intravenously injected in group B, and ketorolac tromethamine injection (0.3 mg/kg) was intravenously injected in group C. The patients in groups A, B, and C were all diluted to 10 mL with normal saline. The control group was in group D, and 10 mL 0.9% normal saline was injected intravenously. Anesthesia induction began 10 minutes later, 0.05 mg/kg midazolam, 4 *μ*g/kg fentanyl, 0.2 mg/kg etomidate, and 0.15 mg/kg cisatracurium. Anesthesia was maintained with 4–8 mg/(kg h) propofol and 0.1–0.2 *μ*g/(kg min) remifentanil. The depth of anesthesia and dosage of muscle relaxants were adjusted according to the surgical requirements. Tracheal intubation was performed after consciousness disappeared. Anesthesia was maintained with propofol 4–8 mg/(kg·h) and remifentanil 0.1–0.2 *μ*g/(kg min) according to the requirements of surgery to adjust the depth of anesthesia and muscle relaxants' dosage. Propofol was stopped at the end of pneumoperitoneum, and remifentanil was stopped at the end of operation. After the patient recovered to spontaneous breathing and swallowing reflex and was able to complete the mandatory response, the tracheal catheter was pulled out. Patient-controlled analgesia was not performed in all groups. If the patients felt unbearable pain after operation and required analgesics, they would receive intramuscular injection of 50 mg pethidine. If satisfactory results are still not achieved, the experiment would be excluded and other analgesic methods would be chosen.

### 2.3. Observation Indicators

1. The mean arterial pressure (MAP) and heart rate (HR) changes at each time point during the quiescent state (T1), immediately intubation (T2), immediately catheter removal (T3), and 5 min after catheter removal (T4) of the four groups were recorded.
2. The changes of visual analogue scale (VAS) and Bruggemann comfort scale (BCS) in the four groups were observed, evaluated, and recorded at 1, 6, 12, and 24 h after operation. The VAS scoring criteria were as follows: 0 point (no pain), 10 points (the most pain), <3 points (good analgesia), and ≥5 points (poor analgesic effect). The BCS scoring criteria were as follows: grade 0 indicates continuous pain, level 1 means it is painless when lying down quietly and aggravating when breathing deeply or coughing, level 2 means that the patient is in a supine and quiet position without pain and has slight pain when taking deep breaths or coughing, level 3 indicates deep breathing without pain, and level 4 means no pain when coughing.
3. Serum tumor necrosis factor-*α* (TNF-*α*), interleukin-6 (IL-6), C-reactive protein (CRP), blood glucose (CLU), and cortisol levels of the four groups before and 6, 12, and 24 h after operation were measured by ELISA.
4. Adverse reactions and additional analgesia of each group within 24 h after operation were recorded.

## 3. Statistical Method

All data were analyzed by SPSS19.0 statistical software, and measurement data were expressed as mean±standard deviation. One-way analysis of variance was used for comparison between groups, and repeated measures analysis of variance was used for comparison at different time points. The count data were expressed as the rate (%) using the *χ*2 test. *P* < 0.05 indicated that the difference was statistically significant.

## 4. Result

### 4.1. Comparison of General Data among Four Groups

There were no significant differences in age, body weight, ASA classification, or the doses of remifentanil and propofol between the four groups (*P* > 0.05), as shown in Table 1.

### 4.2. The MAP and HR Changes of T1, T2, T3, and T4 among Four Groups

The MAP levels of T2, T3, and T4 in the four groups were higher than those of T1, and the HR level was lower than that of T1. The differences were statistically significant (*P* < 0.05). The MAP and HR levels of T2, T3, and T4 in patients of groups A, B, and C were lower than those of group D in the same period (*P* < 0.05). There was no significant difference between groups A, B, and C (*P* > 0.05), as shown in Figure 1.

### 4.3. The VAS and BCS Changes at 1, 6, 12, and 24 h after Operation among Four Groups

The VAS and BCS scores in groups A, B, and C at 1, 6, 12, and 24 h after operation were better than those in group D at the same time, and the differences were statistically significant (*P* < 0.05). The VAS and BCS scores in group A were better than those in groups B and C in the same period at 1 h and 6 h after operation, and the differences were statistically significant (*P* < 0.05). The VAS and BCS scores in groups A, B, and C at 12 h and 24 h during the same period showed no significant difference (*P* > 0.05), as shown in Figure 2.

### 4.4. The TNF-*α*, IL-6, and CRP Changes before Operation and at 6, 12, and 24 h after Operation among Four Groups

Serum TNF-*α*, IL-6, and CRP levels of the four groups at 6, 12, and 24 h after operation were higher than those before operation, and the differences were statistically significant (*P* < 0.05). The levels of serum TNF-*α*, IL-6, and CRP in groups A, B, and C at 6, 12, and 24 h after operation were lower than those in group D. The levels of serum TNF-*α*, IL-6, and CRP in group A at 12 h and 24 h after operation were higher than those in groups B and C, and the differences were statistically significant (*P* < 0.05). The differences in the levels of serum TNF-*α*, IL-6, and CRP at the same time points, i.e., 6, 12, and 24 h after operation, between groups B and C were not statistically significant (*P* > 0.05), as shown in Figure 3.

### 4.5. The CLU and Serum Cortisol Changes before Operation and at 6, 12, and 24 h after Operation among Four Groups

The levels of CLU and serum cortisol in the four groups of patients at 6, 12, and 24 h after operation were significantly higher than those before operation (*P* < 0.05). The CLU and serum cortisol levels in groups A, B, and C at 6, 12, and 24 h after operation were significantly lower than those in group D (*P* < 0.05). The levels of CLU and serum cortisol in group A were lower than those in groups B and C at 6 and 12 h after operation (*P* < 0.05). There was no significant difference in CLU and serum cortisol levels between groups B and C at 6, 12, and 24 h after operation (*P* > 0.05), as shown in Figure 4.

### 4.6. Comparison of Adverse Reactions and Additional Analgesia among the Four Groups

There was no significant difference in the incidence of adverse reactions within 24 h after operation among the four groups (*P* > 0.05). The incidence of additional analgesia in groups A, B, and C was lower than that in group D, and the differences were statistically significant (*P* < 0.05), as shown in Figure 5.

## 5. Discussion

Comfort care is an important part of medical work at present. In recent years, minimally invasive surgery has developed rapidly and significantly reduced the trauma of the operation [9]. Laparoscopic surgery, as a newly developed minimally invasive surgery, has gradually replaced the traditional open surgery. Minimally invasive laparoscopic surgery has many advantages, such as less trauma, shorter time, and faster recovery. Although the trauma is small, postoperative patients may still experience different degrees of pain [10, 11]. The postoperative pain of gynecological laparoscopic surgery was moderate, mainly including incision pain, inflammation and spasm pain of pelvic viscera and tissues, and neck and shoulder pain caused by diaphragmatic traction and lifting caused by carbon dioxide pneumoperitoneum to stimulate phrenic nerves. At the same time, the residual carbon dioxide in abdominal cavity after surgery could be converted into carbonic acid, which caused the body's inflammatory response to the continuous stimulation of peritoneum to aggravate abdominal pain [12–14].

It has important clinical significance to reduce or avoid pain in patients after gynecological laparoscopic surgery. In clinical practice, in order to relieve postoperative pain and inflammation, analgesic measures are usually taken before the injury acts on the body. This treatment is clinically called pre-emptive analgesia [15]. Oxycodone, as an opioid *μ* and *κ* double receptor agonist, took effect 2 min after intravenous injection and peaked at 5 min, lasting for about 3.5 h, without causing histamine release and bradycardia, or inhibiting the parasympathetic nerve, thus exerting a better inhibitory effect on visceral pain [16, 17]. Although pentazocine is an opioid analgesic, its mechanism of action is quite different from morphine. Pentazocine selectively excites *κ* receptor, which is distributed in the brain, brain stem, and spinal cord, thus producing spinal cord analgesia, sedation, and mild respiratory depression. Pentazocine also had a certain excitatory effect on *σ* receptor, but an antagonistic effect on *μ* receptor, so it exerted good analgesic effect, and its respiratory inhibition was lower than that of morphine [18]. Tromethamine is a nonselective and nonsimplified anti-inflammatory drug, which blocks the synthesis of prostaglandins by blocking cyclooxygenase (COX)-1 and COX-2. Ketorolac tromethamine has a strong analgesic effect and is convenient to use. It can be injected intravenously or intramuscularly, has no tolerance in the acute phase, and has no inhibitory effect on respiration, circulation, and central nervous system [19].

The results of this study showed that MAP and HR levels in patients who used oxycodone, pentazocine, and tromethamine for preemptive analgesia during the operation were more stable than those of patients in group D who used normal saline, which suggested that pre-emptive analgesia could effectively relieve the increase of blood pressure and heart rate caused by extubation of endotracheal intubation during the operation. The results of this study also showed that patients who used oxycodone, pentazocine, and ketorolac tromethamine for preemptive analgesia had better VAS and BCS scores as well as serum TNF-*α*, IL-6, CRP, and other inflammatory factor levels in group D at 1, 6, 12, and 24 h after operation. In addition, the VAS and BCS scores of patients who used oxycodone for preemptive analgesia were better than those who used pentazocine and tromethamine ketorolac for pre-emptive analgesia, but the levels of inflammatory factors were higher than those of other two groups. Under normal physiological conditions, various immune factor indicators are in a relatively constant state. When the body receives noxious stimulation, it will enter a stress state, which will activate the hypothalamic-pituitary secretion axis to secrete a variety of neurohormones, thus mediating the increase of proinflammatory factor secretion, causing hyperalgesia and aggravating inflammatory reactions [20]. Oxycodone acts on *μ* receptor and *κ* receptor and has rapid effect, high bioavailability, and analgesic effect for up to 4 hours. It can effectively inhibit postoperative pain and reduce the release of inflammatory factors by reducing the level of cAMP *in vivo* [21]. Oxycodone is more effective in relieving postoperative pain than pentazocine and ketorolac tromethamine. Compared with oxycodone, pentazocine and ketorolac tromethamine can better control the postoperative inflammatory response, but the analgesic and anti-inflammatory effects of pentazocine and ketorolac tromethamine are not different.

After the operation trauma, the body is in a state of stress and the secretion of glucocorticoid increases, which can lead to immunosuppression, pain sensitivity, and delayed recovery. The increased concentration of GLU and cortisol after operation indicated that besides nerve conduction regulating stress response, local inflammatory response was also related to cytokine release. Therefore, a variety of measures were taken to reduce stress response after surgery [22, 23]. The results of this study showed that preoperative analgesia could effectively reduce stress state of patients and oxycodone could effectively inhibit stress response. Studies have shown that oxycodone can promote the release of IL-10, maintain the balance of cytokines, resist proinflammatory cytokines, and better relieve postoperative inflammatory reaction [24].

Gynecological laparoscopic surgery has been widely used in clinical practice, but the incidence of postoperative nausea and vomiting and postoperative pain is high. How to relieve postoperative pain, reduce postoperative nausea and vomiting, and get good postoperative recovery is a very debatable issue. Postoperative pain and irritation of drainage tube and urinary catheters can cause restlessness in the recovery period, resulting in severe consequences such as bleeding at the surgical site, suture rupture of incision, and urinary retention. Analgesic and sedative drugs are commonly used in clinical practice to relieve pain and reduce postoperative restlessness, but they are easy to cause respiratory depression, postoperative nausea and vomiting, and other complications [25]. Studies have shown that pentazocine has less effect on the gastrointestinal tract than morphine and causes less nausea and vomiting [26]. Tromethamine ketorolac has a good analgesic effect, but it also has potential side effects, such as blood coagulation and allergy. It should be disabled when patients have hemorrhagic diseases, gastrointestinal pain, asthma, or liver dysfunction [27]. There was no significant difference in the incidence of adverse reactions within 24 h after operation among the four groups in this study. The incidence of extra analgesia in patients taking oxycodone, pentazocine, and tromethamine for pre-emptive analgesia was lower than that in group D who took normal saline. It indicated that pre-emptive analgesia with oxycodone, pentazocine, and ketorolac tromethamine did not significantly increase postoperative adverse reactions of patients and could effectively reduce the occurrence of additional analgesia.

## 6. Conclusion

Oxycodone, pentazocine, and ketorolac tromethamine are all used for gynecological laparoscopic pre-emptive analgesia, which can effectively inhibit postoperative pain and the generation of inflammatory factors and relieve inflammatory state with good safety. Oxycodone has better postoperative analgesic effect because it can effectively alleviate stress reaction.

## Figures and Tables

**Figure 1:** The MAP and HR changes of T1, T2, T3, and T4 among four groups.

**Figure 2:** The VAS and BCS changes at 1, 6, 12, and 24 h after operation among four groups.

**Figure 3:** The TNF-*α*, IL-6, and CRP changes before operation and at 6, 12, and 24 h after operation among four groups.

**Figure 4:** The CLU and serum cortisol changes before operation and at 6, 12, and 24 h after operation among four groups.

**Figure 5:** Comparison of adverse reactions and additional analgesia among the four groups.

**Table 1:** Comparison of general data among four groups.

Group	Age (years)	Body weight (kg)	ASA classification (I/II)	Remifentanil (*μ*g)	Propofol (mg)
Group A (*n* = 16)	38.92 ± 4.59	58.96 ± 8.16	13/3	816.59 ± 31.42	407.16 ± 16.93
Group B (*n* = 16)	39.05 ± 5.02	59.13 ± 8.85	11/5	821.47 ± 30.94	401.28 ± 18.06
Group C (*n* = 16)	38.75 ± 5.13	60.25 ± 9.04	12/4	813.59 ± 28.73	412.57 ± 19.05
Group D (*n* = 16)	39.16 ± 4.76	59.46 ± 8.74	13/3	819.64 ± 29.94	403.94 ± 17.81
*F*	0.021	0.069	0.958	0.209	1.168
*P*	0.996	0.976	0.811	0.889	0.329

## Data Availability

Data are available on request to the authors.
